The article "Molecular Mechanisms of Antifungal Resistance in Mucormycosis" was published in 2022. Journal: Biomed Res Int.

# Molecular Mechanisms of Antifungal Resistance in Mucormycosis

**DOI:** 10.1155/2022/6722245

**Published:** 2022-10-13

**Authors:** Priya Ganesan, Dhanraj Ganapathy, Saravanan Sekaran, Karthikeyan Murthykumar, Ashok K. Sundramoorthy, Sivaperumal Pitchiah, Rajeshkumar Shanmugam

**Affiliations:** ^1^Department of Prosthodontics, Saveetha Dental College and Hospitals, Saveetha Institute of Medical and Technical Sciences, Chennai, India; ^2^Department of Periodontics, Saveetha Dental College and Hospitals, Saveetha Institute of Medical and Technical Sciences, Chennai, India; ^3^Nanobiomedicine Lab, Department of Pharmacology, Saveetha Dental College and Hospitals, Saveetha Institute of Medical and Technical Sciences, Chennai, India

## Abstract

Mucormycosis is one among the life-threatening fungal infections with high morbidity and mortality. It is an uncommon and rare infection targeting people with altered immunity. This lethal infection induced by fungi belonging to the Mucorales family is very progressive in nature. The incidence has increased in recent decades owing to the rise in immunocompromised patients. Disease management involves a multimodal strategy including early administration of drugs and surgical removal of infected tissues. Among the antifungals, azoles and amphotericin B remain the gold standard drugs of choice for initial treatment. The order Mucorales are developing a high level of resistance to the available systemic antifungal drugs, and the efficacy still remains below par. Deciphering the molecular mechanisms behind the antifungal resistance in Mucormycosis would add vital information to our available antifungal armamentarium and design novel therapies. Therefore, in this review, we have discussed the mechanisms behind Mucormycosis antifungal resistance. Moreover, this review also highlights the basic mechanisms of action of antifungal drugs and the resistance landscape which is expected to augment future treatment strategies.

## 1. Introduction

Emerging number of fungi linked to illnesses in humans, animals, and plants is increasing, thanks to developments in molecular methods and phylogenetic analyses, which have led to a better understanding of fungal taxonomy and the creation of new dangerous fungi [1]. Aggressive fungal infections are rare since the body's immune system is capable of destroying large organisms, but they can be difficult for clinicians to treat, especially in severely ill individuals and patients who are immunocompromised as a result of disease or immunosuppressive medications. Infections produced by fungi can cause high mortality rates in some patients, particularly those who are immunocompromised or critically unwell. Invasive fungal infections are difficult to treat because eukaryotic pathogens' medication target sites are very similar to those of the human host, limiting therapy options [1].

Antifungals belong to many pharmacological classes that target various biological processes, either fungistatic or fungicidal the pathogenic yeast's growth. The creation of the cell wall, cytoplasmic membrane, and RNA biogenesis are among these biological activities, biosynthetic routes involving a series of enzymes. The pharmacokinetics of medications is a significant element that influences drug efficacy [2]. Factors such as drug metabolism, intake, and distribution can all have an impact on a medicine's effectiveness. Furthermore, treatment efficacy is affected by the severity of the illness as well as the size of the infecting organisms' population. Antifungal drugs' efficacy in the treatment of fungal infections may be influenced by differences in drug bioavailability between various tissues. Azole medications' bioavailability is much lower in low-pH vaginal tissues than in the blood. Importantly, the tissue distribution and toxicity of different lipid formulations differ [3].

Biofilms can be formed on the surfaces of medical equipment such as catheters by fungi. These biofilms appear to be resistant to antifungal penetration and may have fewer therapeutic targets. Successful therapies rely heavily on the human immune system. Antifungal medications, azoles, in particular, rely on the immune system of the host to treat invasive fungal infections [3, 4]. Antifungal medication resistance of the infected species is another key aspect that can lead to therapeutic failure.

In long-term usage of azole medications such as fluconazole, for example, it is possible that pathogenic yeasts will develop resistance to it, rendering the therapy ineffective. Fluconazole is the most commonly prescribed azole for fungal infection prevention and treatment. However, azole resistance has emerged in a number of species, which is a new concern that is generating therapeutic failures [5].

## 2. Mucormycosis

Mucormycosis is a fatal infection caused by fungi of the Mucoromycotina subfamily and Mucorales order, which belong to a group of lower fungi previously known as zygomycetes and are a phylogenetically archaic group of microorganisms. The groups Rhizopus, Mucor, Lichtheimia, Cunninghamella, Rhizomucor, and Apophysomyces are among the causative agents of mucormycosis [6]. The group contains a variety of widely dispersed ancestral lineages in the fungal tree of life. Mutations are thought to have accumulated over time. The opportunistic Mucorales are divided into the families Cunninghamellaceae, Lichtheimiaceae, Mucoraceae, Saksenaceae, and Syncephalastraceae, with Mucoraceae and Lichtheimiaceae causing the vast majority of human infections. Rhizomucor was shown to be outside the Mucoraceae family in the molecular phylogenetic analysis [7].

Mucormycosis outbreaks have been found in wards, among victims of disasters like the Joplin disaster, and among soldiers recovering from combat-related injuries, circinelloides-related foodborne outbreaks in healthy people, illustrate Mucorales' propensity to cause serious illnesses.

It has become more common in hematologic malignancies and organ transplantation as the condition is the second most prevalent mould infection, and it is also becoming more common in people with uncontrolled diabetes or ketoacidosis. Despite rigorous antifungal treatment, in certain, significant surgical debridement, mucormycosis-related mortality remains unacceptably high [8].

A recent report shows an increase in a number of activity of mucormycosis in COVID-19 patients. It can damage the sinuses, brain, or lungs and is thus fairly prevalent in patients who have COVID-19 or are recovering from it [9] Swelling on one side of the face, fever, headache, nasal or sinus congestion, and black lesions on the nasal bridge or upper inside of the mouth are all common signs of mucormycosis (Table 1).

## 3. Antifungal Drugs

Antifungals belong to many pharmacological classes that target various biological processes, either fungistatic or fungicidal pathogenic yeast's growth. The production of the cell wall, cytoplasmic membrane, and RNA biogenesis are among these biological activities, biosynthetic routes involving a series of enzymes [14] (Figure 1).

## 4. Mechanism of Action of Antifungal Drugs

### 4.1. Targeting Ergosterol Biosynthesis

Ergosterol is the most abundant sterol in fungal cell membranes, especially plasma and mitochondria. In the cell membrane, sterols and sphingolipids combine to generate lipid rafts. Lipid rafts contain bioactive proteins including those involved in signaling, stress response, breeding, and nutrition transport. The structure of these membranes is critical for fungi to survive. A cascade of 25 enzymes catalyzes the manufacture of ergosterol. Because ergosterol is an essential lipid for fungus and plants, but not for humans, this metabolic pathway is a good target for medicines [15]. There are various groups of drugs that effects the biosynthesis of ergosterol mechanisms such as the azoles, polyenes, allamines, and morphines. The most prevalent antifungal medicine class used to treat fungal infections is azoles. Azoles inhibit the enzyme 14–demethylase (Erg11p), which is involved in the production of ergosterol. Azoles attach to Erg11p, thereby lowering ergosterol levels in cells. When Erg11p is blocked, subsequent enzymes in the pathway (Erg6p, Erg25p, Erg26p, Erg27p, and Erg3p) produce a fungistatic poisonous sterol; azoles are also responsible for increasing reactive oxygen species levels (ROS). The infecting fungus' development is inhibited by both high ROS levels and harmful sterol synthesis [16].

Whereas the polyene antifungal drugs attack the ergosterol within the cell membrane. It creates pores when they bind to ergosterol. Monovalent ions (K+, Na+, H+, and Cl) seep quickly through pores, resulting in fungal cell death. Amphotericin B and nystatin are polyene medicines; however, amphotericin B is still utilized for systemic treatment [17]. In the allylamine group of drugs, squalene epoxidase in the ergosterol production is the target of these antifungals. Terbinafine (Lamisil), flunarizine, and naftifine are examples of these medications. Terbinafine (Lamisil) is a drug that is frequently used to treat dermatophyte infections [18]. Fenpropimorph, tridemorph, and amorpholine are all examples of morphines. Ergosterol biosynthesis C-14 sterol reductase is the target (Erg24p). Morpholines are widely employed in agriculture, but they are extremely harmful to people. Nail dermatophyte infections are treated with a 5% amorolfine hydrochloride-containing nail lacquer solution [19]. In addition to conventional antifungal agents, medicinal plants are also widely explored against fungal pathogens. The aqueous extract of Tulbaghia violacea acquired by maceration exhibits antifungal activity by decreasing the production of ergosterol which negatively impacted lipid production in Aspergillus flavus [20]. Deciphering the mechanism behind this action, it was found that the enzyme oxidosqualene cyclase was mainly targeted by the extract which led to the accumulation of 2,3-oxidosqualene.

### 4.2. Targeting Cell Wall Biosynthesis

The fungal outer wall has a stiff exterior covering, and it serves as the initial line of protection against osmotic stress. Because mammalian cells lack cell walls, enzymes in cell wall synthesis are the main targets. Echinocandin antifungal drugs such as caspofungin, micafungin, and anidulafungin target the cell wall [21]. They act on the enzyme 1-3 glucan synthase, which is encoded by three genes: FKS1, FKS2, and FKS3. The 1-3 glucan synthase enzyme is a three-protein complex (Fks1p, Fks2p, and Fks3p) that uses UDP-glucose to synthesize 1-3-glucan, a key component of the fungal cell wall. These drugs are often fungicidal and are generally chosen due to their low human toxicity [22]. To date, antifungal agents have been developed for inhibiting the cell wall component biosynthesis. Poacic acid inhibits *β*-1,3-glucan synthesis, breaking its integrity by inhibiting the activity of Gas and Crh enzymes involved in cell wall remodeling [23]. It was found to modulate and affect the regulatory mechanisms involved in rescue responses.

Owing to the selectively targeting of fungal cell wall, echinocandins do not exert their activity on mammalian cells. High specificity reduced the off targeted effects and adverse events with echinocandin use in comparison to other antifungal drugs such as azoles and amphotericin B [24]. In a randomized double-blinded study, caspofungin (50 mg) has no adverse drug reactions in HIV-infected patients treated for esophageal candidiasis [25]. In contrast, its use in invasive candidiasis and aspergillosis was associated with infrequent reports of hepatotoxicity and nephrotoxicity [26, 27]. The safety of caspofungin in 1205 patients with daily doses ranging from 35 to 100 mg exhibited no dose-related adverse effects and toxicity [28]. Surprisingly, even at higher doses (150 mg/day), no adverse effects were observed in patients with invasive candidiasis [29]. In treatment for invasive candidiasis, caspofungin showed excellent safety profile without any drug-related side effects [30]. Interestingly, a clinical trial evidenced high safety and efficacy in immunocompromised paediatric patients [31]. Similar to caspofungin, micafungin also was found to be safe in both adult and pediatric population. In pediatric patients, it was well tolerated with only 4.7% patients experiencing serious side effects [32]. A multicentrer, randomized, open-label study (Phase III) investigating the prophylactic use of micafungin (50 mg/day) along with itraconazole in neutropenic patients with haemotopoietic stem cell transplantation demonstrated no drug-related adverse effects. In addition, it was found to be safer in prevention of fungal infections invasion compared to intraconazole [33]. In allogenic haematopoietic stem cell transplantation procedure, micafungin was found to be safe with only 1.4% discontinuation [34]. In *Candida* infections, patients with daily dose (50 mg, 75 mg, and 100 mg) of anidulafungin and follow-up study indicated no dose-dependent adverse effects and only 9.0% deaths were reported in highly complicated and comorbid patients [35]. A prospective, multicenter study in critically ill patients following various clinical conditions and candidaemia, invasive candidiasis, anidulafungin IV therapy accounted to only 1.9% of severe adverse effects. In the pediatric population, 0.75 mg/kg and 1.5 mg/kg per day dose of anidulafungin was associated with no adverse effects and well tolerated by children. Overall, these reports indicate that echinocandins is safe and well-tolerated profiles were observed in adult and pediatric patients [36].

### 4.3. Targeting the Synthesis of RNA and DNA

5-Flucytosine (5FC) prevents the formation of nucleic acids. The cytosine permease enzyme is used by sensitive cells to import 5FC. 5FC is metabolized to 5FU, which is then transformed to 5-fluorouridine triphosphate. Rather than uridine triphosphate, 5FUTP is integrated into fungal RNA, altering protein translation. 5FU can also be transformed to 5-fluorodeoxyuridine monophosphate (5FdUMP), which inhibits thymidylate synthase, a key enzyme in DNA biosynthesis [37].  Figure 2 shows the mechanism of actions.

## 5. Mechanism Antifungal Drug Resistance

### 5.1. Azole Drug Resistance

Azoles inhibit ergosterol biosynthesis by actively targeting cytochrome P450-dependent enzyme, lanosterol 14-*α*-demethylase. Ergosterol biosynthesis inhibition leads to the intracellular accumulation of toxic intermediates which perturbs the membrane stability and arrests fungal growth [38]. Resistance to azole antifungals has also been linked to the overexpression of 14-*α*-demethylase. In Aspergillus and Candida resistance strains, overexpression/alteration in *ERG11/cyp51A/cyp51B* was observed with substitutions in amino acid residues proximal to the heme-binding site of 14-*α*-demethylase [39]. Constitute expression of *ERG11* owing to a gain-of-function mutation in the Upc2, a transcriptional activator confers azole resistance to C. *albicans [*40*]*. C. glabrata transcription factor (TF) CgRpn4 was found to be responsible for azole resistance by reducing fluconazole accumulation and regulating the membrane permeability [41]. Candida also develops azole resistance by mutating *ERG11*. In a recent report, Set1 mediates the H3K4 histone methylation and loss of SET1 increases susceptibility to azoles by affecting *ERG11* expression [42]. In addition to this, *ERG3* mutations results in ergosterol depletion or alternative sterols accumulation and this depends on three stress response regulatory proteins including molecular chaperone Hsp90, protein phosphatase calcineurin, and protein kinase C1 [43].

Overexpression of cytochrome P450 enzymes is another route adopted to confer resistance to azoles. Researchers investigated the azole-resistant C. glabrata isolate and discovered that it had a higher ergosterol content. In-depth investigations portrayed a higher microsomal P450 levels leading to increased ergosterol synthesis in the resistance strain and was responsible for both azole and amphotericin B resistance [44]. These findings indicate that the cross-resistance to such two triazoles was caused by elevated P450 levels [45]. In the small number of clinical isolates with 14 *α*-demethylase overexpression, this phenomenon was only seen in C. glabrata, and the possibility that other resistance mechanisms are active in the same strain all suggests that increased expression of the target enzyme ends up playing just a minor role in clinical azole resistance [46].

Resistance to antifungal agents is also conferred by overexpression of multidrug transporters, alteration of drug target, and the initiation of stress responses. Pathogenic yeast contains a considerable number of membrane proteins which are located in the cell membrane, vacuolar surface, and mitochondrial membrane. [47]. They are involved in environmental sensing, nutrient transport, signal transduction, drug efflux, drug alteration, and drug detoxification processes. For instance, membrane protein found in the mitochondrial membrane Atm1p, an ABC transporter, is involved in iron homeostasis, whereas Mlt1p, a membrane transporter found at the vacuolar membrane, transports phosphatidylcholine [48]. A solitary membrane carrier can perform a variety of physiological tasks. Azole resistance has been linked to two forms of membrane transporters found in fungi [49]. ABC-Ts (adenosine triphosphate binding cassette transporters) are ATP-dependent active transporters. Each ABC-T is made up of two lattice domains (MSD) with six transmembrane sections and each two nucleic acid binding domains. Each NBD has an ABC (ATP-binding cassette), which binds ATP [50]. Major facilitator transporters (MFS-T) require a gradient of protons in the cytoplasm as an energy source in order to transfer xenobiotics. MFS-Ts have 12 to 14 transmembrane segments and lack the NBDs that define ABC-Ts [51]. The pleiotropic drug resistance transporter (PDR) belonging to the ABC transporters was found to be tightly associated with drug resistance. In *Mucor circinelloides*, out of the eight *pdr* genes, pdr1 and pdr2 was found to be involved in the resistance towards isavuconzaole, ravuconazole, and posaconazole [52] According to a comparison of fluconazole accumulation by C. albicans and C. krusei [53], all research strains accumulated the same amount of fluconazole in the first 60 minutes. C. krusei, on the other hand, collected 60% less fluconazole after 90 minutes of incubation than C. albicans, demonstrating that active efflux is implicated in the fluconazole sensitivity of these C. krusei strains.

The rise of resistance to azoles by various fungal species has worsened the landscape of treating several fungal diseases. Azole derivatives such as azole-triphenylphosphonium conjugates have shown to alleviate drug resistance in *Candida* strains by interfering with mitochondrial functions and while retaining the ability to inhibit ergosterol biosynthesis [54]. As most azole drugs exhibit their activity by targeting Erg11, by mining the existing repository of chemical compounds, new compounds targeting Erg 11 are explored to combat antifungal resistance. A 2,5-disubstituted pyridine compound CpdLC-6888 was found to inhibit Erg 11 similar to conventional azole drugs [55].

### 5.2. Polyene Drug Resistance

Resistance to polyene drugs like amphotericin B, and nystatin is unusual, but resistant isolates have been found. Polyene resistance is linked to changes in ERG3 and ERG6. In fungal strains, disrupting ERG3 and ERG6 causes decreased ergosterol concentrations and amphotericin B sensitivity in vitro [56]. One of the major mechanisms behind resistance is the polyene-induced reduction in oxidative stress [57]. Apart from this, altered sterol composition of the membrane was also found to induce resistance to AmB in *A. terrus* [57]. A catalase-dependent mechanism is more likely to be involved in the resistance of counteracting oxidative stress induced by AmB [58].

Candida auris exhibits resistance to amphotericin B and the underlying mechanism depicted alterations in membrane lipids and in chromatin modifications. More importantly, increased phosphorylated MKc1 cell integrity MAP kinase in response to AmB treatment was found to be a major resistance pathway behind the resistance [59]. Another mechanism behind the AmB resistance was found to be the involvement of heat shock proteins Hsp70 and Hsp90, key players in governing cellular stress. Three plausible mechanisms were proposed behind the acquisition of AmB resistance: (1) Hsp90 disruption would lead to the generation and endurance of new genetic variations, (2) Hsp90 may chaperone various cell signaling regulators to augment the development of new adaptive phenotypes, and (3) active Hsp90 would regulate the stabilization of several mutated cell regulators which have the tendency to induce AmB resistance [60]. Other mechanisms behind the AmB resistance are reviewed extensively [61]. Fryberg proposed that resistance occurs as a result of the selection of sources of resilient cells, which are present in small proportions throughout the population. These naturally resistant cells create sterols with a decreased affinity for nystatin. The usual growth rate as well as the rate at which nystatin destroys the cell membrane dictate the rate of growth in the presence of nystatin. The affinity of nystatin for membrane sterols is hypothesized to influence the rate of membrane damage: the greater the nystatin-sterol affinity, the greater the rate of membrane damage [62]. The biochemical notion that resistance develops as a result of changes in the sterol contents of the cells, either quantitatively or qualitatively, resistant cells with lower sterol content bind fewer polyene than sensitive cells. This reduced polyene binding in C. albicans mutants could be attributable to a drop in the cell's total ergosterol concentration without corresponding changes in sterol composition, or the replacement of some or all of the polyene-binding sterols with ones that bind polyene less tightly [63]. Other studies show a relationship between the polyene employed to isolate mutants and cross-resistance, as well as the selection of mutants with specific pol gene mutations. The wild type had the most ergosterol and dehydroergosterol, according to sterol analysis of the parent and mutations. The latter sterol, on the other hand, was absent in the pol2 mutant and only present in trace amounts in the pol3 mutant. Though the relationship between pol genes is unknown, evidence from UV spectroscopic analysis revealed that these mutants act in sequence rather than parallel, showing that they are epistatically linked [64] (Figure 3).

## 6. Possible Approaches to Tackle Antifungal Resistance in Mucormycoses

Mucorales are very destructive and cause lethal infections (Mucormycosis) in patients with altered immunity and predisposing conditions. The international treatment guidelines for mucormycosis involve amphotericin B as a first-line treatment strategy and posaconazole is followed as salvage therapy [65]. However, fungi are now intrinsically resistant to these routinely used drugs which narrow down the choice of drugs. For instance, a very unique mechanism through which *Mucor circinelloides* confers resistance to rapamycin and antifungal agents FK506 is by epimutation [66]. RNAi-based silencing of the genes targeted by the drug for short period and reexpression following drug passage is the causative mechanism behind the resistance [52]. This transient epimutation observed requires in-depth elucidations to unravel the mechanisms and develop novel approaches to combat drug resistance. Besides this, monotherapies using a single drug would be surpassed with a combinatorial therapeutic strategy involving multiple antifungal drugs in a phased manner. Mouse models of diabetes and neutropenic infected with *R. arrhizus* showed improved survival upon combined treatment with an echinocandin and a polyene rather than monotherapy [67]. Synergistic interactions between L-micafungin, AmB, and an iron chelator deferasirox showed higher efficiency against Mucorales fungi in diabetic rats [68] Micafungin inhibits fungal efflux pumps and upon combined administration with azole which enhances the intracellular uptake and retention [69]. Furthermore, in a study in patients with rhinocerebral mucormycosis, a combination of caspofungin and a polyene improved survival [70]. Thus, it is clear that combinatorial therapy is superior to the use of a single antifungal agent which results in the development of drug resistance.

Another strategy to negate antifungal drug resistance is therapeutic drug monitoring in patients. The development of drug resistance at high doses and off-targeted effects can also be minimized by maximizing the therapeutic potential through the aforementioned approach. Futuristic investigations are needed to delineate the mechanisms of tolerance and resistance. In vitro simulations and model predictions by utilizing the available pharmacokinetic data will aid in developing drugs with safer therapeutic doses. Integrated pharmacodynamics and pharmacokinetic approaches will aid in the identification of drug concentrations with maximum kill kinetics and reduction in antifungal resistance [71]. Truncated knowledge of Mucorales physiology and its molecular mechanisms of pathogenesis also dampens the development of new antifungals. The critical question of how to stem the rise of antifungal resistance can be addressed in the forthcoming years by involving next-generation sequencing and functional genomics to better identify the virulence determinants.

An extensive understanding of mucormycosis necessitates the use of animal models which portray/simulate all possible comorbidities, but they usually fail to recapitulate exact clinical scenarios.

## 7. Future Directions and Conclusions

Mucormycosis is a pathogen that the host's immune system suppresses in the microbiota. As it becomes one of the widespread infections among the immunocompromised patients and the therapeutic index is variably decreasing due to multidrug resistance more research is needed to gain a better knowledge of these mechanisms of action and resistance, which could help with the detection of resistant isolates and the development of novel pharmacological targets would aid in the prevention of drug resistance. The continuous upsurge in COVID-19 cases with mucormycosis could favor clinical evaluation strategies for early diagnosis and better evaluate the resistance scenario. It is noteworthy to understand that there is a huge gap in the comprehensive validation of drugs across all the members of Mucorales. Therefore, there is a pressing need to involve promising molecular tools for in-depth evaluation and reducing mortality by combating antifungal resistance. The inclusion of CRISPR-Cas technology will aid in deciphering the antifungal resistance mechanisms and untie the knots due to genetic intractability. Another area for futuristic investigations is to understand the interactions between Mucorales and macrophages. Species-specific differences are observed in the killing of Mucorales spores by macrophages which would add to the resistance landscape. Therefore, disseminating the cellular scenarios facilitating the survival of Mucorales inside the macrophage will expand the knowledge to develop effective treatments against this lethal infection. Overall, appropriate treatment modules at an early stage are essential to decrease the mortality rate in mucormycosis. Additional investigations are essential to delineate the molecular mechanisms of resistance and its role in vivo owing to the inability to correlate in vitro data with clinical outcomes.

## Figures and Tables

**Figure 1:** Targets of antifungal drugs.

**Figure 2:** Mechanism of actions of antifungal drugs.

**Figure 3:** Mechanism of antifungal drug resistance.

**Table 1:** Antifungal drugs used in mucormycosis.

Commonly used antifungal drugs in mucormycosis		
Target mechanism of action in the pathogen	Antifungal drugs	Reference
Ergosterol biosynthesis	Azoles	[10, 11]
	Polyenes	
	Allylamines	
	Morphine	
Cell wall biosynthesis	Echinocandins	[12]
Nucleic acid synthesis	5-Flucytosine	[13]

## Data Availability

The data used in this study were done by the authors.
